The article "Investigation on Inorganic Salts K2TiF6 and KBF4 to Develop Nanoparticles Based TiB2 Reinforcement Aluminium Composites" was retracted in 2023. Reasons: signs of a paper mill; suspected computer-generated content; unreliable results or conclusions; concerns about the data.

# Investigation on Inorganic Salts K2TiF6 and KBF4 to Develop Nanoparticles Based TiB2 Reinforcement Aluminium Composites

**DOI:** 10.1155/2022/8559402

**Published:** 2022-01-30

**Authors:** Vinayagam Mohanavel, K. Ravi Kumar, T. Sathish, Palanivel Velmurugan, Alagar Karthick, M. Ravichandran, Saleh Alfarraj, Hesham S. Almoallim, Shanmugam Sureshkumar, J. Isaac JoshuaRamesh Lalvani

**Affiliations:** ^1^Centre for Materials Engineering and Regenerative Medicine, Bharath Institute of Higher Education and Research, Selaiyur, Chennai 600073, Tamil Nadu, India; ^2^Department of Mechanical Engineering, KPR Institute of Engineering and Technology, Coimbatore-641407, Tamilnadu, India; ^3^Department of Mechanical Engineering, Saveetha School of Engineering, SIMATS, Chennai 602 105, Tamil Nadu, India; ^4^Department of Electrical and Electronics Engineering, KPR Institute of Engineering and Technology, Coimbatore 641407, Tamil Nadu, India; ^5^Department of Mechanical Engineering, K. Ramakrishnan College of Engineering, Tiruchirappalli-621112, Tamilnadu, India; ^6^Zoology Department, College of Science, King Saud University, Riyadh 11451, Saudi Arabia; ^7^Department of Oral and Maxillofacial Surgery, College of Dentistry, King Saud University, PO Box-60169, Riyadh-11545, Saudi Arabia; ^8^Department of Animal Resources Science, Dankook University, 119,Dandae-ro, Cheonan,31116, Republic of Korea; ^9^Department of Mechanical Engineering, Faculty of Mechanical and Production Engineering, AMIT, Arbaminch University, Ethiopia

## Abstract

In the current research, AA6082 aluminium alloy matrix composites (AAMCs) incorporated with various weight fractions of titanium diboride (0, 3, 6, and 9 wt%) were prepared via an in situ casting technique. The exothermic reaction between inorganic powders like dipotassium hexafluorotitanate (K2TiF6) and potassium tetrafluoroborate (KBF4) in molten Al metal contributes to the development of titanium diboride content. The manufactured AA6082-TiB2 AAMCs were evaluated using a scanning electron microscope (SEM) and X-ray diffraction (XRD). The mechanical properties and wear rate (WR) of the AAMCs were investigated. XRD guarantees the creation of TiB2 phases and proves the nonappearance of reaction products in the AMCs. SEM studies depict the even dispersion of TiB2 in the matrix alloy. The mechanical and tribological properties (MTP) of the AAMCs showed improvement by the dispersion of TiB2 particles. The WR decreases steadily with TiB2 and the least WR is seen at nine weight concentrations of TiB2/AA6082 AAMCs. Fabricated composites revealed 47.9% higher flexural strength and 14.2% superior compression strength than the base AA6082 alloy.

The article "Investigation on Inorganic Salts K2TiF6 and KBF4 to Develop Nanoparticles Based TiB2 Reinforcement Aluminium Composites" was retracted in 2023. Reasons: signs of a paper mill; suspected computer-generated content; unreliable results or conclusions; concerns about the data.

## 1. Introduction

In recent scenarios, a huge number of research studies has shifted from monolithic materials to composite materials to meet the improving universal demand for high performance, ecofriendly corrosion, erosion, and wear-resistant materials. The improvement of lightweight and fewer costly materials with enriched performance for automobiles, construction, aviation, aircraft, and several engineering applications is always a concern of numerous research workers [1, 2]. The foremost goal involved in developing composite (AMC) materials is to merge the ductile matrix metals and hard ceramic particles. AAMCs have enormous potential in being tailored for several applications and are qualified for replacing conventional materials. Some of the good-locking properties of AAMCs comprise superior specific strength, excellent elastic modulus, and excellent specific stiffness in comparison with their monolithic alloy [3–5].

The AAMCs are broadly manufactured through the liquid state route. The liquid state processing method may be of two types: ex situ (stir casting technique) and in situ (direct melt reaction technique or exothermic salt-metal reaction technique) fabrication [6–8]. The in situ process exhibits even scattering of particles [9]. The type of filler or reinforcement material significantly influences the MTP of the AMCs. Titanium diboride (TiB_2_) is an ultrahigh temperature ceramic particle with good covalent bonding, providing it with a high melting temperature of 3225°C, a higher Vickers hardness of 3400 HV, and a low density of 4.5 g/m3. Moreover, in contrast to most ceramics, TiB2 reveals good thermal shock confrontation and superior electrical and thermal conductivity [10, 11]. Tjong and Lau [12] developed Al-4%Cu/TiB_2_ AAMCs through the hot isostatic pressing method and found that the hardness and yield strength enriches with the inclusion of TiB_2_ filler material. Natarajan et al. [13] achieved a dry sliding wear test on an AA6063 composite strengthened with in situ TiB_2_ content and observed that the inclusion of harder ceramic TiB_2_ enriches the MTP of the proposed AAMCs. Christy et al. [14] carried out their research on aluminum alloy AA6061/TiB_2_ AMCs, where the TiB_2_ filler contents were made through the magneto chemistry exothermic reaction of halide powders in the Al melt at 840^o^C and examined the microstructural and mechanical behavior of the composites. Rajasekaran and Sampath [15] produced AA2219/TiB_2_ in situ AMCs synthesized through an exothermic reaction process at 800^o^C employing KBF_4_ and K_2_TiF_6_ inorganic salts. SEM micrograph examination exhibited the hexagonal shape of in situ TiB_2_ particle content. Ramesh et al. [16] produced AA6061/TiB_2_ AAMCs through an exothermic reaction process and analyzed the tensile strength (UTS) of the AMCs. Wang et al. [17] synthesized A356/TiB_2_ AAMCs by in situ reaction of flux powders in liquefied aluminum and noticed that the UTS and YS of AAMCs increased with a rise in TiB_2_ particles. Rajan et al. [18] prepared AA7075/TiB_2_ AAMCs through the magneto chemistry reaction of halide powders to liquefied aluminum and described that the inclusion of filler content in AMCs enriches the wear protection and enhances the tribological characteristics. The tribological behavior of AA6061 base aluminium and AAMCs reinforced with diverse mass concentrations of titanium diboride was analyzed by Shobha et al. [19] and Suresh et al. [20]. Poria et al. [21] evaluated the impact of TiB_2_ particle content on the MTP of LM4/TiB_2_ AMCs. The SEM images of the worn surface analysis reveal the hybrid mode of wear mechanisms. The presence of TiB_2_ acts as a hindrance to the movement of dislocations that causes high wear resistance compared to the unreinforced alloy. Pazhouhanfar and Eghbali [22] observed that AA6061/TiB_2_ composite matrix microstructure refinement was better in comparison with the unreinforced monolithic alloy prepared by the melt stirring route. The mechanical characteristics of AAMCs are boosted incrementally by the rise in TiB_2_ particle weight concentration.

The article "Investigation on Inorganic Salts K2TiF6 and KBF4 to Develop Nanoparticles Based TiB2 Reinforcement Aluminium Composites" was retracted in 2023. Reasons: signs of a paper mill; suspected computer-generated content; unreliable results or conclusions; concerns about the data.

AA6082 (aluminum alloy) is a thermal-treatable moderate-strength alloy for architectural and transport applications because of its outstanding formability, machining capacity, welding capacity, and superior corrosion resistance. In AA6082 alloys, vast quantities of magnesium regulate the grain structure, rendering it even at higher temperatures, which makes it highly proficient. It was observed that not much work was carried out on the mechanical, tribological, and microstructural characterization of the AA6082 alloy with TiB_2_ reinforcement particle content. The principal target of this study is to establish an in situ composite material reinforced with TiB_2_. The microstructures, fractured and worn surfaces of the developed AAMCs samples were examined using SEM and XRD. Hence, the present study aims to manufacture the in situ casting method and examine the role of TiB_2_ particles as well as the weight fraction of tensile strength (UTS), hardness, compression strength (CS), wear rate (WR), and flexural strength (FS) of the composite.

## 2. Experimental Work

### 2.1. Manufacturing of AA6082/TiB2 AAMCs

Aluminum alloy (AA6082) was used in this work as the material matrix and the AAA6082 chemical constituents are displayed in Table 1. The AA6082 alloy in rod shape was melted using a melting furnace with a graphite crucible. Table. 2 shows the properties of the AA6082 aluminium.  Figure 1 displays the casting furnace arrangement.

The article "Investigation on Inorganic Salts K2TiF6 and KBF4 to Develop Nanoparticles Based TiB2 Reinforcement Aluminium Composites" was retracted in 2023. Reasons: signs of a paper mill; suspected computer-generated content; unreliable results or conclusions; concerns about the data.

The gauged quantities of chemicals are revealed in Table 3 which were incorporated into the molten AA6082 to form TiB_2_ (0. 3, 6, and 9 wt%). If we increase the appropriate % wt to greater than 10% in situ, it leads to large-sized blow holes and castings that will be brittle in nature. To prevent Al_3_Ti formation, KBF_4_ halide powder was marginally higher than the stoichiometric ratio. The melting temperature was held at 850°C. The AA6082/TiB_2_ melt was constantly stirred at 400 rpm and held for 1800 sec. The AA6082/TiB_2_ AAMC thaw was poured into a preheated mould and composite samples were obtained.

### 2.2. Microstructure and Testing

The essential dimension of the specimens was cut from the synthesized castings. The test samples were refined as per a standard metallographic procedure. The microstructure was witnessed utilizing an SEM. XRD spectrums were documented by a Panalytical X-ray diffractometer. Applying a load of 0.5 Kgf for a dwell interval of 15 s, Vicker's hardness test has measured the microhardness. The hardness was tested at six different places, and the mean hardness value was determined for the sample.

Figure 2(a) displays the fabricated tensile specimens. Tensile tests were performed as per ASTM using a computerized UTM. The tensile samples were processed by measuring the length of forty mm, the width of seven mm, and the thickness of six mm. Four tests and the mean values have been recorded in each combination. In compliance with ASTM E9 standards, the compression strength (CS) was borne in the UTM. The compression test specimens have also been manufactured in cylinder forms of 8 mm in diameter and 24 mm in height. The specimens machined from the synthesized AAMCs were machined and polished metallographically. The specimens after the compression test are exposed in Figure 2(b). Flexural tests were achieved on the AA6082 parent material and the prepared AAMCs using the computerized UTM.

Using a DUCOM TR20-LE pin on the disc (POD) wear testing unit, wear resistance was assessed at room temperature in dry wear conditions as per the ASTM G99-04 standard. The POD system schematic diagram is presented in Figure 2(c). The test sample is made from AA6082 alloy and is a manufactured composite of diameter 8 mm and length 32 mm. After extensive washing using acetone solvent, the specimen was measured using an automated measuring system before and after the sliding wear test. Initial and final weight disparities resulted in mass loss due to sliding wear. The WR was assessed employing the following relation:

(1) $$\begin{array}{c} W=\frac{M}{\rho \;D}, \end{array}$$

where *W* is the WR (mm^3^/m), *M* is weight loss (g), *ρ* is density (g/mm^3^), and *D* is the rotating distance (*m*). The pin surface was polished and the end of the pin was attached to a hard steel disc (62 HRc). Testing was carried out with the usual forces of 10N, 20N, and 30N and a sliding speed of 1 m/s at sliding distances of 1500 m. The samples before the wear test are illustrated in Figure 2(d).

The article "Investigation on Inorganic Salts K2TiF6 and KBF4 to Develop Nanoparticles Based TiB2 Reinforcement Aluminium Composites" was retracted in 2023. Reasons: signs of a paper mill; suspected computer-generated content; unreliable results or conclusions; concerns about the data.

## 3. Results and Discussion

### 3.1. SEM Analysis of AA6082/TiB_2_ AAMCs

Figure 3(a) illustrates the SEM images of the base AA6082 alloy. The microstructure of AA6082 alloy exposes the occurrence of magnesium (Mg) and silica (Si) content in AA6082 alloy. Figure 3 depicts the SEM micrograph of the AA6082/TiB2 AAMCs. Figures 3(b)–3(f) show the SEM photograph of AA6082/TiB2 AMCs that exhibit the dissemination of TiB2 contents in the Al material. Microstructural examination proves the homogeneous dissemination of TiB2 filler content in the AA6082 alloy and also exhibits a strong attachment between the secondary and primary material. The SEM photograph presented in Figures 3(e) and 3(f) shows the stable and pure interface between the parent metal and TiB2 filler content. The Al matrix-TiB2 particle interface indicates a high level of interface consistency between the AA6082 matrix and the reinforcement without reaction product presence. The homogeneous dissemination of reinforcement particles is more essential to enrich the mechanical properties of the AA6082. These results are in line with the earlier studies by several researchers [16].

### 3.2. XRD Analysis of AA6082-TiB2 AAMCs

Figure 4 depicts the XRD spectrums of the AA6082 alloy and TiB_2_ AAMCs. The XRD plot demonstrated the presence of respective elements of aluminium and TiB_2_ particles in the prepared composites and also, the pattern reveals the absence of reaction products.

XRD spectrums guarantee the existence of aluminum (in the most prominent peaks) and TiB_2_ (revealed by minor peaks) in the AAMCs. With a rise in the mass concentration of TiB_2_ in the AAMCs, the amplitude of the peaks of TiB_2_ improved [10, 13]. The prepared composites' aluminum peaks are slightly higher than the AAMCs, as shown in Figure 4. In the composites, no other unwanted compounds were discovered. The thermodynamically stable TiB2 particles can be ensured.

### 3.3. Hardness

The microhardness (MH) of the AA6082/TiB_2_ AAMCs is exposed in Figure 5. The MH increases with a rise in TiB_2_ particles. The test outcomes reveal the enrichment in MH of the AA6082/TiB2 AAMCs from 51 HV to 87 HV. The enrichment in MH could be attributed to even allocating TiB_2_ in the Al matrix [13]. The accretion of TiB_2_ content in the AA6082 matrix improves the surface area, thereby reducing the matrix's grain size. Aluminium alloys with 9 wt% of TiB_2_ composites exhibit superior hardness. It can be ascribed to the enriched surface area of the TiB_2_ contents that presents huge protection to plastic deformation (PD), which directs to raise the MH of AAMCs.

The article "Investigation on Inorganic Salts K2TiF6 and KBF4 to Develop Nanoparticles Based TiB2 Reinforcement Aluminium Composites" was retracted in 2023. Reasons: signs of a paper mill; suspected computer-generated content; unreliable results or conclusions; concerns about the data.

Other researchers showed similar forms of findings in their analysis. The AA6061/AlN AMCs are due to the grain alteration of the matrix (Hall–Petch mechanism) and the impact of particulate matter on the Orowan strengthening of AAMCs, according to Ashok Kumar and others [23].

Even the strong AlN secondary materials act as barricades against dislocation movement, thereby increasing the hardness of the composite in contrast with the monolithic Al alloy. Ravi Kumar et al. [24] noted that the rise in hardness of the composites AA6063/TiC with 10wt% of TiC has more robust plastic resistance. Rajeswari et al. [25] have identified the effects on the hardness and UTS of the AAMCs of stirring speed, mass concentration, and processing temperature. Mathan Kumar et al. [26] have observed that because PD decreases by the strengthening particles, adding AlN, ZrB_2_, and Si_3_N_4_ particles increased the hardness of AMCs. The strength of the AA6082/TiB_2_ AMCs then increased to an overall 70.58% and 9% of TiB_2_.

### 3.4. Tensile Strength of AA6082/TiB_2_ AAMCs

Figure 6 illustrates the influence of TiB_2_ particles on the UTS of the AAMCs. The UTS of the fabricated AAMCs was augmented from 176 MPa to 201 MPa. The UTS of the composite was originated to be higher at 9 wt% TiB_2_ content. Such kinds of escalation were stated by other investigators while incorporating SiO_2_ [27], rice husk ash [28], eggshell [29], nanosilver [30], basalt [31], AlN [32], and WC [33] particles in AMCs. Although the incorporation of graphite [34], SiC [35, 36], coconut shell ash [37], and mica [38] particles declined the UTS of the AAMCs.

The following can be clarified as the critical reasons behind the enrichment of the AA6082/TiB_2_ AMC in UTS. The penetration of secondary TiB_2_ material into the matrix results in many dislocation densities in solidification around the reinforcing particles. This is due to a missuit between the soft matrix AA6082 and the hard TiB_2_ secondary material, caused by the coefficient of thermal expansion. As well as the thermal missuit between matrix and reinforcement, upshots are often introduced to enhance the load-bearing capacity of strong reinforcing particles that enrich the strength of composites [15, 20].

The article "Investigation on Inorganic Salts K2TiF6 and KBF4 to Develop Nanoparticles Based TiB2 Reinforcement Aluminium Composites" was retracted in 2023. Reasons: signs of a paper mill; suspected computer-generated content; unreliable results or conclusions; concerns about the data.

Tensile strength is enriched to a maximum of 14.20% while incorporating 9% of TiB_2_. A similar trend of outcomes was revealed by other investigators in their study. Gopalakrishnan and Murugan [39] noticed the appreciable enrichment in the UTS of the AA6061/TiC AAMCs. Pardeep Sharma et al. [40] reported that the sound integrity closeness between the Si_3_N_4_/graphite contents and the AA6082 alloy augmented the UTS of the AAMCs. Jebeen Moses et al. [41] have described the influence of blade angle, stirring speed, and stirring time on the hardness and UTS of the AAMCs. Shalaby and Churyumov [42] observed that the load transfer between the hard AlNp and soft matrix A359 alloy results in strengthening and improved tensile strength. Sivananth et al. [43] exhibited that the UTS and fatigue strength of AAMCs were enhanced with augmenting TiC particles, and the occurrence of TiC particles in AAMCs serves as an obstruction to dislocation, thereby enriching the UTS of the AMC. This kind of intensifying factor enhances the rise in the inclusion of TiB_2_ particles. The direct mechanism achieved the strengthening of AMCs, precisely the escalation in PD of the AAMCs and the secondary mechanism, specifically the thermal misfit between the liquid matrix and solid reinforcement [18, 23].

### 3.5. Tensile Fracture Surface Analysis of AA6082/TiB_2_ AAMCs

Figure 7 depicts the tensile fracture morphology of AA6082/TiB_2_ AAMCs. The fracture of the monolithic alloy shows ductile fracture with bigger size dimples, as shown in Figure 7(a). Figures 7(b)–7(d) show that the inclusion of TiB_2_ content significantly diminishes the quantum of dimples. The participation of incorporated content in the parent alloy steadily changes the mode of failure between ductile fractures and brittle and ductile fractures. A significant number of flat areas are located on the AA6082/TiB_2_ AAMCs fracture area, which reveals sufficiently high brittle fracture and minor ductile fracture. Figure 7(d) indicates a tremendous number of broken reinforcing particles on the fracture site, which allows for superior interfacial connections between the matrix and strengthening contents [18, 20]. A similar form of findings was revealed by other investigators in their analysis. Tian et al. [44] described that the fractography exhibits strong evidence of sound attachment between the matrix and the secondary materials leading to enriching the UTS of the AAMCs. Thangarasu et al. [45] noticed that the uniformly distributed bigger-sized voids occurred in the fracture surface of the AA6082 alloy which reveals that ductile rupture is the principal fracture mechanism. Dinaharan et al. [46] expressed the tensile fractography of AA6061/10 wt% of ZrB_2_p composites exhibiting smaller size dimples compared to that of AA6061 alloy. Karbala Akbari et al. [47] noted that the presence of the solid nature of the filler materials in the composites reduces the formation of voids.

The article "Investigation on Inorganic Salts K2TiF6 and KBF4 to Develop Nanoparticles Based TiB2 Reinforcement Aluminium Composites" was retracted in 2023. Reasons: signs of a paper mill; suspected computer-generated content; unreliable results or conclusions; concerns about the data.

### 3.6. Compression Strength of AA6082/TiB_2_ AAMCs

The impact of TiB_2_ on the CS of the AA6082/TiB_2_ composite is displayed in Figure 8. The CS was observed to enhance with the rise of TiB_2_, and it is extremely superior to the CS of the unreinforced monolithic alloy. The occurrence of brittle and hard TiB_2_ particles in the matrix works as a hindrance for the dislocation movement that enriches the CS of the AA6082/TiB_2_ AAMCs. Thus, the CS of the AAMCs is drastically enhanced. The CS reaches peak values at 9 wt% of TiB_2_ particles in the AA6082 base alloy. The important reason for the enhancement in the CS of AAMCs is the occurrence of the solid nature of TiB_2_ particles in the soft matrix which resists the PD during compressive load. Superior compression strength may be owed to the strengthening impact of the TiB_2_ contents. Moreover, the enhancement in the sound connection between the AA6082 and TiB_2_ contents improves the compression strength. This outcome is in decent agreement with the upshot of Sajjadi et al. [48]. Baradeswaran et al. [49] and Auradi et al. [50] have ensured that up to 20 wt% B_4_C particles and up to 7 wt% B_4_C particles' compression strength is enhanced, notably with an increase in weight fraction of boron carbide.

### 3.7. Flexural Strength of the AA6082/TiB_2_ AAMCs

The influence of TiB_2_ particles on the flexural strength (FS) of AA6082/TiB_2_ AMCs is shown in Figure 9. The FS of AAMCs was boosted steadily with an escalation in the weight concentration of TiB_2_ content in the matrix. The magnificent enhancement in FS of AAMCs is obtained at 9 wt% TiB_2_ particles in the AA6082 matrix. This can be mainly ascribed to the conveying of the applied load from the soft matrix to the hard nature of TiB_2_ particles. Enhancement in FS is also owing to the superior mechanical attachment between the TiB_2_ and the AA6082 alloy. Hence, the value of FS at 9 wt% of TiB_2_/AA6082 composites exhibits superior results as compared to monolithic alloys. The even dispersion of TiB_2_ in the AMCs offered more protection to the PD of the AMCs which was intended to enhance the flexural strength. Normally, the addition of TiB_2_ content upshots in a significant increase in composite strength, and the enrichment in flexural strength of the AMCs was due to the enhanced particle weight percentage of the AMCs. A similar enrichment is also stated by the investigator Mohanavel et al. [51] for the AA6351/AlN AAMCs.

The article "Investigation on Inorganic Salts K2TiF6 and KBF4 to Develop Nanoparticles Based TiB2 Reinforcement Aluminium Composites" was retracted in 2023. Reasons: signs of a paper mill; suspected computer-generated content; unreliable results or conclusions; concerns about the data.

### 3.8. Effect of TiB_2_ in the AA6082 Matrix on WR

The influence of TiB_2_ content on the WR of AA6082/TiB_2_ AAMCs is illustrated in Figure 10. The AA6082/9 wt% TiB_2_ AMCs have the least WR compared to the AA6082 base alloy. Enrichment of wear resistance in the AA6082/TiB_2_ AMCs is not only owing to the occurrence of TiB_2_ particles that serve as load-bearing elements but also to refinement in grain size. The strong mechanical bonding between the AA6082 matrix and the TiB_2_ particle content impedes the removal of particles during the wear test [13, 20]. Therefore, the WR gradually decreases with an escalation in TiB_2_ wt% of filler particles. Figure 10 shows the WR of the composite is 5.865 × 10^−3 ^mm^3^/m which is lower than the matrix AA6082. Moreover, the hardness of the materials is inversely proportional to the WR as per Archard's theory. Because the augment in hardness of the composite enhances the resistance to sliding wear. Basavarajappa et al. [52] examined the effect of rotating speed on the wear characteristics and revealed the subsurface deformation of composites. Michael Rajan et al. [53] noticed that the WR of the composite enhances steadily with the escalation in load for all temperature ranges utilized. The WR enriches with the increase in normal load and declines with an increase in the weight fraction of TiB_2_. Soorya Prakash et al. [54] stated that the inclusion of rock dust particles to the AA6061 alloy enriched the wear protection of the AAMCs. Moses et al. [55] observed that the wear resistance of the AAMCs was enhanced with an increase in the weight percentage of TiCp. Also, the hard TiC contents include the plain matrix, which helps to decrease the PD affected by the improved wear resistance of the composite.

Figure 10 indicates the influence of applied load (AL) on the WR of the parent alloy and AA6082/TiB_2_ AMCs. The figure reveals that the WR enhances with intensifying AL and at all the load conditions, with the minimum wear rate found to be 9 wt% TiB_2_/AA6082 AMCs. The frictional heat (FH) that is generated on the contact surface increases with the applied load. This softens the matrix material. A superior degree of material shifting between the counter surfaces takes place. A movement to subsurface deformation and minor cracking enhances with augmenting the applied load. The enriched wear rate is also influenced by massive quantum of particle fragmentation. The applied load influences the region of interaction between the counter surfaces. The contact level controls the magnitude of the heat generated by friction. Thus, the asperities in the steel disks on the surface of the softened pin contribute to increased WR speeds. In addition, the wear protection of the composites at all loads considered was higher than that of the parent alloy.

The article "Investigation on Inorganic Salts K2TiF6 and KBF4 to Develop Nanoparticles Based TiB2 Reinforcement Aluminium Composites" was retracted in 2023. Reasons: signs of a paper mill; suspected computer-generated content; unreliable results or conclusions; concerns about the data.

### 3.9. Worn Surface Analysis of AA6082/TiB_2_ AMCs

The impact of TiB_2_ content on the morphology of the worn surfaces (WS) of AA6082/TiB_2_ composites is illustrated in Figure 11(a). It is detected from the figure that the worn surface of the AA6082 alloy reveals a huge quantum of plastic flow (PF) of the matrix alloy. FH is generated between the surface of the rotating pin and the counter steel disc which induces plasticity along with the matrix. The wear mode appears to be adhesive. In Figures 11(b)–11(d), the worn surfaces of the AA6082/TiB_2_ composite exhibit occurrence of shallow grooves and a few pits. The occurrence of TiB_2_ particles opposes the PF of material during wear testing [6, 22]. A mild level of PF is noticed at the boundaries of the grooves. The PF of the WS is minimized, and distinct multiple grooves like shapes start to form (Figure 11)(d) as the weight proportion of TiB_2_ is enhanced to 9 wt%. Moreover, the delicate and parallel grooves are visible along the direction of sliding. The TiB_2_ particle proposes opposition to the mobility of the plasticized matrix and diminishes the contact surfaces. Thus, equivalent forms of grooves are formed as the wear mode progressively transfers from adhesive to abrasive. It is additionally seen from the figure that, due to the inclusion of TiB_2_ in the matrix, the debris is loose but not adherent to it.

## 4. Conclusions

In the current investigation, AA6082/TiB2 AMCs were developed by the salt-metal reaction technique, and the following conclusions were derived:

1. The AA6082 alloy AMCs strengthened with 0, 3, 6, and 9 wt% of TiB2 content were effectively prepared by the in situ method.
2. The SEM micrograph reveals the homogeneous dispersion of TiB2 content in the AA6082 alloy, and the XRD plots guarantee the existence of TiB2 in the produced AMCs.
3. The UTS of the AAMCs was boosted from 176 MPa to 201 MPa with the accumulation of TiB2 particles.
4. AA6082/TiB2 AAMC tensile fractures demonstrate a hybrid fracture mode, i.e., a brittle and ductile fracture mode.
5. Flexural strength and compression strength augments drastically with the rise in TiB2 particle content. Composites exhibited 47.9% superior flexural strength and 14.2% higher compression strength compared to the monolithic AA6082 alloy.
6. The WR decreases linearly with the addition of TiB2, and the minimum WR is obtained at a 9 weight percentage of TiB2. The enhanced weight of TiB2 particulates altered the abrasive wear characteristic from adhesion.
7. The inclusion of TiB2 particles into the AA6082 matrix has shown a great enrichment in the mechanical and wear behavior of the AAMCs.
8. The synthesized TiB2 content exhibited several morphologies like hexagonal, spherical, and cubic structures.

The article "Investigation on Inorganic Salts K2TiF6 and KBF4 to Develop Nanoparticles Based TiB2 Reinforcement Aluminium Composites" was retracted in 2023. Reasons: signs of a paper mill; suspected computer-generated content; unreliable results or conclusions; concerns about the data.

## Figures and Tables

**Figure 1:** Stir casting furnace.

**Figure 2:** (a) Tensile test samples. (b) Compression test samples. (c) Schematic illustration of tribometer. (d) Wear samples.

**Figure 3:** SEM micrographs of AA6082/TiB_2_ AAMCs with TiB_2_ content. (a) 0 wt%, (b) 3 wt%, (c) 6 wt%, (d) 9 wt%, and (e, f) 9 wt% (higher magnification).

**Figure 4:** XRD patterns of the produced AA6082/TiB_2_ composites.

**Figure 5:** Impact of hardness on the wt% of TiB_2_ particles.

**Figure 6:** Influence of tensile strength on the wt% of TiB_2_ particles.

**Figure 7:** SEM microphotographs of tensile fracture surfaces of AA6082/TiB_2_ AMCs with TiB_2_ content. (a) 0 wt%, (b) 3 wt%, (c) 6 wt%, and (d) 9 wt%.

**Figure 8:** Influence of compression strength on the wt% of TiB_2_ particles.

**Figure 9:** Influence of flexural strength on the wt% of TiB_2_ particles.

**Figure 10:** Wear rate with varying applied load for AA6082 and AA6082/TiB_2_ composites.

**Figure 11:** SEM micrographs of the worn surface of (a) 0 wt% TiB_2_, (b) 3 wt% TiB_2_, (c) 6 wt% TiB _2_, and (d) 9 wt% TiB_2_.

**Table 1:** Chemical constituents of AA6082 aluminum.

Element	Si	Fe	Mn	Mg	Ti	Al
Weight (%)	1.0	0.60	0.5	0.7	0.20	Bal

**Table 2:** Characteristics of AA6082 aluminum.

Sl. no.	Properties	
1	Density	2.71 g/cm^3^
2	UTS	140–330 MPa
3	YS	90–280 MPa
4	Ductility	14%
5	Hardness	40 HB
6	Proof stress	85 MPa

**Table 3:** The calculated weights of inorganic salts.

TiB_2_ (wt%)	0	3	6	9
K_2_TiF_6_ (grams)	0	104	207	311
KBF_4_ (grams)	0	131	262	391

## Data Availability

The data used to support the findings of this study are included in the article. Further data or information required are available from the corresponding author upon reasonable request.
